RETRACTED

# Butyrate Attenuates Lipopolysaccharide-Induced Inflammation in Intestinal Cells and Crohn's Mucosa through Modulation of Antioxidant Defense Machinery

**DOI:** 10.1371/journal.pone.0032841

**Published:** 2012-03-06

**Authors:** Ilaria Russo, Alessandro Luciani, Paola De Cicco, Edoardo Troncone, Carolina Ciacci

**Affiliations:** 1 Department of Clinical and Experimental Medicine, Federico II University of Naples, Napoli, Italy; 2 Department of Chemical Engineering, University of Naples “Federico II”, Naples, Italy; 3 Chair of Gastroenterology, University of Salerno Medical School, Baronissi, Italy; Charité-University Medicine Berlin, Germany

## Abstract

Oxidative stress plays an important role in the pathogenesis of inflammatory bowel disease (IBD), including Crohn's disease (CrD). High levels of Reactive Oxygen Species (ROS) induce the activation of the redox-sensitive nuclear transcription factor kappa-B (NF-κB), which in turn triggers the inflammatory mediators. Butyrate decreases pro-inflammatory cytokine expression by the lamina propria mononuclear cells in CrD patients via inhibition of NF-κB activation, but how it reduces inflammation is still unclear. We suggest that butyrate controls ROS mediated NF-κB activation and thus mucosal inflammation in intestinal epithelial cells and in CrD colonic mucosa by triggering intracellular antioxidant defense systems. Intestinal epithelial Caco-2 cells and colonic mucosa from 14 patients with CrD and 12 controls were challenged with or without lipopolysaccaride from *Escherichia Coli* (EC-LPS) in presence or absence of butyrate for 4 and 24 h. The effects of butyrate on oxidative stress, p42/44 MAP kinase phosphorylation, p65-NF-κB activation and mucosal inflammation were investigated by real time PCR, western blot and confocal microscopy. Our results suggest that EC-LPS challenge induces a decrease in Gluthation-S-Transferase-alpha (GSTA1/A2) mRNA levels, protein expression and catalytic activity; enhanced levels of ROS induced by EC-LPS challenge mediates p65-NF-κB activation and inflammatory response in Caco-2 cells and in CrD colonic mucosa. Furthermore butyrate treatment was seen to restore GSTA1/A2 mRNA levels, protein expression and catalytic activity and to control NF-κB activation, COX-2, ICAM-1 and the release of pro-inflammatory cytokine. In conclusion, butyrate rescues the redox machinery and controls the intracellular ROS balance thus switching off EC-LPS induced inflammatory response in intestinal epithelial cells and in CrD colonic mucosa.

## Introduction

Intestinal epithelial cells constitute the interface between the gut lumen and the innate and adaptive immune system [1]. Previous studies show that a loss of immunologic tolerance is the primary cause for the development of inflammatory bowel disease (IBD) in genetically susceptible hosts [1], [2].

RETRACTED

IBD is characterized by the loss of tolerance in the intestinal immune system towards the intestinal microbiota resulting in constant immune activation which leads to mucosal tissue damage and chronic inflammation [3]. These spontaneously relapsing chronic intestinal inflammations are subdivided into two main idiopathic pathologies ulcerative colitis (UC) and Crohn's Disease (CrD).

CrD is characterized histologically by transmural inflammation, epithelial ulceration, fissure formation, and stenosis of segments throughout the gastrointestinal tract [4]. Increased ROS production and decreased antioxidant enzyme levels have been found in the intestinal mucosa of CrD patients [5], [6], causing increased oxidative stress, lipid peroxidation and inflammation [7], [8]. Moreover high ROS levels have been reported to promote activation and translocation of NF-κB [9] into the nucleus through alternative phosphorylation of Iκ-B-α which leads to its ubiquitynation and degradation [9]. This ROS/NF-κB self-sustaining regulatory loop may contribute to the perpetuation and exacerbation of chronic inflammation [10].

CrD therapy is presently based on anti-inflammatory non-steroid drugs such as mesalazine, steroid analogues, and/or immuno-suppressive molecules that often produce severe side-effects [11]. An emerging therapeutic approach is the use of specific dietary fibre and/or prebiotics able to enhance butyrate production in the colon of CrD patients [12]. These functional foods have proven effective in delivering butyrate to the colonic mucosa, a process that is difficult to achieve by direct administration of butyrate, either orally or rectally [13]. Butyrate is a four-carbon short-chain fatty acid produced by bacterial fermentation of mainly undigested dietary carbohydrates within the colonic lumen. Although butyrate has been the favoured energy source for colonic epithelial cells and induces changes in gene expression influencing colonic function [14],[15], it has recently been demonstrated to have an anti-inflammatory effect [16]. In two in vitro studies, butyrate was shown to modulate inflammation through NF-κB inhibition [17] and up-regulation of PPAR-γ [18]. Several in vivo studies report a decreased inflammation after rectal administration of butyrate or mixtures of SCFA (short chain fatty acids) in patients with active ulcerative colitis [19],[20] and diversion colitis [21],[22]. However, the detailed biological regulatory mechanisms of butyrate's activity remain unclear.

Since the impaired mucosal anti-oxidative capacity may further promote intestinal inflammation in patients with IBD [23], this study aimed to investigate whether butyrate could modulate GST-A1/A2 mRNA levels, protein expression and catalytic activity and readjust ROS levels, thus switching off ROS mediated NF-κB activation and the inflammatory response in intestinal epithelial Caco-2 cells and CrD colonic mucosa.

RETRACTED

## Materials and Methods

### Patients and ex-vivo organ cultures

Biopsy specimens were taken from uninflamed mucosal areas immediately next to inflamed tissues of fourteen patients with CrD (n = 14, mean age 24 years, range 18–41). The primary site of involvement was ileal in four patients, ileocolonic in four and colonic in five. Disease was active in all patients, as defined by a Crohn's Disease Activity Index (CDAI) of >150 [24]. Normal controls (n = 12, mean age 22.4 years, range 18–29) included mucosal samples taken from eight patients with uncomplicated diverticular disease and four patients with rectal bleeding due to haemorrhoid. Informed written consent was obtained from all subjects, and the protocol of the study was approved by the Ethics Committee of Regione Campania Health Authority. One specimen from each patient was used for diagnosis; the other samples were cultured in vitro for 4 and 24 h [25] with medium alone, EC-LPS (1 µg/ml E. Coli Serotype O127: B8 Lipopolysaccharide, Sigma-Aldrich, Milan, Italy) in the presence or absence of the butyrate (10 mM).

### Cell lines

Caco-2 cells, a human colonic epithelial cell line, were cultured as recommended by the American Type Culture Collection (ATCC). Experiments were initiated on day 14 or 15 after seeding and continued for 24–72 h, as the cells progressed through more mature stages of differentiation.

### Cell cultures

Cells were seeded onto 12-well plates at a density of 2–3×10^5^cells/cm^2^ and were pre-treated with butyrate (10 mM) for 24 h and finally stimulated with EC-LPS (1 µg/ml^−1^) for another 4 h and 24 h.

### RNA interference

Cells were seeded onto 12-well plates (Costar®, Corning) at a density of 2–3×10^5^cells/cm^2^. The cells were transfected with human GSTA1/A2 or scrambled small interfering RNA (50 nmol/L, siRNA) duplex using Lipofectamine RNAiMAX at 37°C for 72 h. Cells were then stimulated in the presence of butyrate with EC-LPS for 4 h and 24 h. The GSTA1/A2 duplex siRNA was a pool of two sequences: siRNA no. 1, GSTA1 (catalog number HSS142318, Invitrogen, Milan, Italy) and siRNA no. 2, GSTA2 (catalog number HSS142323, Invitrogen, Milan, Italy)

### Quantitative RT–PCR

Total RNA was extracted using the RNA-easy Mini Kit (Qiagen). The mRNA was reverse transcribed with a SuperScriptTM III First Strand Synthesis System (Invitrogen). Quantitative RT–PCR was performed with an iCycler iQ Multicolour Real-Time PCR Detector (Bio-Rad) with iQ TM SYBR Green supermix (Bio-Rad). Expression levels of genes were normalized to β-actin levels in the same sample. Primer sequences were as follows (5′ to 3′, sense, antisense): GSTA1, Forward primer CCT GCC CAC AGT GAA GAA GT Reverse primer GCC TCC ATG ACT GCG TTA TT; GSTA2, Forward primer GGC TGC AGC TGG AGT AGA GT Reverse primer ATTGGCACTTGCTGGAACAT; β-Actin, Forward primer TGACCCAGATCATGTTTGAG Reverse primer TAATCTCCTTCTGCATCCTG. The relative amounts of mRNA were calculated by using the comparative Ct method.

RETRACTED

### Nuclear protein extraction

The cells were collected in cold buffer A (10 mmol/L HEPES (pH 7.9), 1.5 mmol/L MgCl_2_, 10 mmol/L KCl, and 1 mmol/L dithiothreitol (DTT) and protease inhibitor cocktail), homogenized in Potter-Elvehjem pestle and glass tube (Sigma-Aldrich), and centrifuged at 11,000× g for 20 min at 4°C to obtain nuclear pellets. Supernatants were collected as cytoplasmic fractions. Nuclear pellets were washed with buffer A and resuspended in buffer B (20 mmol/L HEPES (pH 7.9), 1.5 mmol/L MgCl_2_, 0.42 mol/L NaCl, 0.2 mmol/L EDTA, 25% (v/v) glycerol, 1 mmol/L DTT, and protease inhibitor cocktail) and incubated on ice for 50 min with occasional mixing to extract nuclear proteins. Nuclear extracts were cleared by centrifugation (11,000× g, 15 min, 4°C), and supernatants were collected as nuclear fraction. Then, cytoplasmic and nuclear whole-cell fractions were analyzed by immunoblotting.

### Immunoblot

Experiments were carried out as previously described [26]. Briefly, cells were washed in ice-cold phosphate-buffered saline (PBS) and lysed with NP-40 lysis buffer (1% NP-40, 150 mmol/L NaCl, 50 mmol/L Tris, pH 7.4, 10 mmol/L NaMoO_4_) at 4°C for 30 min. Protease inhibitors were added to NP-40 lysis buffer to a final concentration of 1 µg^.^ml^−1^ leupeptin, 2 µg^.^ml^−1^ aprotinin, 50 µg^.^ml^−1^ Pefabloc, 121 µg^.^ml^−1^ benzamidine, 3.5 µg^.^ml^−1^ E64. Cell lysates were centrifuged at maximal speed in an eppifuge at 4°C, and supernatants were collected. Cell lysates (50 µg) were loaded, separated on 10% SDS-PAGE and transferred to nitrocellulose. After blocking for 2 h (TBS/Tween supplemented with 5% nonfat dry milk), blots were incubated with anti-phospho-p65NF-κB(Cell Signaling Technology, Danvers, Massachusetts, USA), Gluthatione-S-transferase α (goat polyclonal IgG, Abcam, Milan, Italy), phospho-p42/p44 MAP kinases (rabbit polyclonal IgG, Cell Signaling Technology), COX-2 (Cell Signaling Technology, Danvers, Massachusetts, USA), ICAM-1 (SantaCruz Biotechnology, Santa Cruz, California, USA) and β-actin (rabbit polyclonal IgG; Santa Cruz, CA, USA) and αβ-tubulin (rabbit polyclonal IgG; Santa Cruz, CA, USA). The primary antibodies were counterstained using a horseradish peroxidase-conjugated anti-IgG antibody (Amersham, Little Chalfont, UK) for 60 min at room temperature. Proteins were visualized by chemiluminescence (ECL Plus, Amersham) and exposed to X-OMAT film (Eastman Kodak, Rochester, NY). Protein concentrations were determined using a Bio-Rad protein assay to ensure equal protein loading prior to Western blot analysis.

RETRACTED

### Immunolocalization

#### Human tissue sections

Five µm thick cryostat sections were fixed in acetone for 10 min. The sections were individually incubated for 2 hours at room temperature with the following antibodies: phopsho-p65NF-κB(Ser536) (rabbit polyclonal; Cell Signaling Technology), p42/p44 MAPK (rabbit polyclonal IgG ; Cell Signaling Technology), COX-2 (rabbit polyclonal; Cell Signaling Technology, Danvers, Massachusetts, USA) and ICAM-1 (rabbit polyclonal; SantaCruz Biotechnology, Santa Cruz, California, USA). Antigen expression and distribution was visualized using a donkey anti-rabbit IgGs conjugated to Alexa Fluor 488 for 60 min at room temperature. Isotype control antibodies (IgG1 or IgG2), isotype-matched non immune Igs, or isotype-matched antibodies against inappropriate blood group antigens were used as control of specificity. Data were analyzed under fluorescence examination using a LSM510 Zeiss confocal laser scanning unit (Carl Zeiss, Germany). COX-2 or ICAM-1 positive mononuclear cells (MNC) were counted per mm^2^ of mucosa. Epithelial cells with nuclear p65 localization were counted per 100 epithelial cells. Data were examined in a blind fashion by two independent reviewers totally unaware of all the culture conditions to prevent bias in their observation [27],[28].

### Measurement of intracellular reduced glutathione (GSH)

Intracellular GSH levels were measured in Caco-2 cells using a fluorometric method as described by Ranganna *et al.* [29]. Briefly, cells were collected in ice-cold NaCl/Pi were pelleted by centrifugation (750 g, 5 min, 4°C). The pellets were suspended in buffer A (50 mL of 25% (w/v) metaphosphoric acid and 188 mL of 0.1 mmol/L sodium phosphate buffer supplemented with 5 mmol/L EDTA, pH 8.0) and homogenized on ice. The homogenates were centrifuged (15,000 g, 20 min, 4°C) and diluted 10-fold with 0.1 mL sodium phosphate buffer B (5 mmol/L EDTA, pH = 8.0) incubated with buffer C (1.8 mL buffer B and 0.1 mL 0.1% o phthalaldehyde solution in methanol ) for 15 min at room temperature. Changes in fluorescence were analyzed with a Wallac 1420 multilabel Counter (PerkinElmer Waltham, MA, USA) at an activation wavelength of 350 nm and an emission wavelength of 420 nm. Cellular GSH levels were calculated using standard curve measurements performed simultaneously with the samples and expressed as pmole of GSH/cell.

RETRACTED

### ROS detection

The cells and five-micrometer cryostat sections were pulsed with 10 µmol/L 5-(and-6)-chloromethyl-2′7′-dichlorodihydrofluorescein diacetate acetyl ester (CM-H2DCFDA) (Molecular Probes, Invitrogen) [26]. CM-H2DCFDA, a ROS-sensitive probe, was used to track changes in the cellular redox state. The cells were analyzed with a Wallac 1420 multilabel Counter (PerkinElmer Waltham, MA,USA) and detected by a LSM510 Zeiss confocal laser scanning unit (Carl Zeiss, Germany).

### ELISA

TNF-α secretion was measured using the BD OptEIATM ELISA kit II (BD Biosciences) according to the manufacturer's instructions. Protein concentrations of whole-cell lysates were measured using the BioRad Dc protein Assay (BioRad). TNF-α levels were normalized to standard protein concentrations [30].

### Statistical analysis

All of the experiments were performed in duplicate and repeated at least three times. Group data from all experiments are presented as means ± s.d. . One-way ANOVA was used for all of the statistical analyses among multiple groups. In another set of data the paired two tailed Student's test was used for statistical analyses. Groups were compared by post hoc Tukey-Kramer test. A probability of *P*-value<0.05 was considered significant.

## Results

### Effect of butyrate on GSTA1/A2 mRNA levels, protein expression and catalytic activity and ROS levels in intestinal epithelial cells upon challenge with LPS from *Escherichia Coli*

We demonstrated that butyrate prevents LPS-induced decrease of GSTA1/A2 mRNA, protein and activity in LPS-stimulated intestinal epithelial cells (Figure 1A and B and Figure S1A). To establish that butyrate induces GST expression in lipopolysaccharide stimulated Caco-2 cells, the influence of an siRNA construct specific to GSTA1/A2 was evaluated. Results showed that butyrate-induced GST-α protein (Figure S1B and Figure 1D) was almost completely silenced when Caco-2 cells were transfected with GST A1/A2 siRNA prior to stimulation with butyrate whereas negative siRNA transfection had no relevant effect on butyrate-induced GST expression (Figure S1B).

**Figure 1:** Effect of butyrate on GSTA1/A2 mRNA levels and protein expression in intestinal epithelial cells and CrD mucosal epithelial cells challenged with LPS from *Escherichia Coli*. (**A–B**) Caco-2 cells were treated for 24 hours with butyrate and then were stimulated with EC-LPS for 4 h. (**A**) Real time PCR of GSTA1/A2 mRNA. Values are means ± s.d., n = 6. Asterisks indicate that means differ from samples cultured with medium alone and from samples cultured with EC-LPS. *P<0.05. (**B**, *top line*) Immunoblot of GST-α. β-actin was used as loading control for blot. (**B**, *bottom line*) Densitometric analysis of the band intensity. Values are means ± s.d., n = 6. (**C–D**) CrD colonic mucosa were cultured for 4 h in the presence of medium alone, medium with EC-LPS or EC-LPS with butyrate. (**C**) Real time PCR of GSTA1/A2 mRNA. Values are means ± s.d., n = 14. Asterisks indicate that means differ from samples cultured with medium alone and from samples cultured with EC-LPS. *P<0.05. (**D**) confocal microscopy of GST-α protein (green) in CrD colonic mucosa (n = 14). Nuclei counterstained with DAPI(blue). Scale bar, 10 µm.

RETRACTED

Using a well established tissue culture model for biopsy of human CrD colonic mucosa [28], we showed that butyrate prevents LPS-induced decrease of GSTA1/A2 mRNA, protein and activity in LPS-treated colonic mucosa in CrD patients (Figure 1C and D and Figure S1C).

Since glutathione-S-transferases (GSTs) play an important role in protection mechanisms against oxidative stress, we investigated the capacity of butyrate-induced GST-α expression to attenuate lipopolysaccharide-mediated oxidative stress in intestinal epithelial cells and CrD colonic mucosa.

We demonstrated that butyrate was effective in controlling the increase of ROS levels and attenuating the concomitant decline in reduced glutathione (GSH) levels generated in response to lipopolysaccharide in intestinal epithelial cells (Figure 2A and Figure S2A). GSTA1/A2 siRNA antagonized the down-regulatory effect of the butyrate on ROS levels and decline in GSH levels induced by EC-LPS (Figure 2A and Figure S2A). We investigated the effect of butyrate in controlling oxidative stress in CrD epithelia. Before challenge, higher ROS levels were observed in CrD colonic mucosa compared with controls. EC-LPS challenge led to an increase of ROS levels at 4 hours of incubation in CrD colonic mucosa but not in controls (Figure 2B). Moreover treatment of cultured biopsies with butyrate was highly effective in preventing LPS-induced ROS levels (Figure 2B).

**Figure 2:** Effect of butyrate on oxidative stress in intestinal epithelial cells and CrD mucosal epithelial cells challenged with LPS from *Escherichia Coli*. Caco-2 cells were treated for 24 h with butyrate or transfected with either 50 nM human GST-α siRNA or scrambled oligonucleotides and then challenged with EC-LPS for 4 h. (**A**) Intracellular ROS levels. Values are means ± s.d., n = 6. Asterisks indicate that means differ from samples cultured with medium alone and from samples cultured with EC-LPS. *P<0.05. [DCF: 2′,7′-dichlorodihydrofluorescein]. (**B**) ROS levels in control (n = 10) and CrD colonic mucosa (n = 14) before challenge and after challenge with medium alone, medium with EC-LPS or EC-LPS with butyrate following 4 h of incubation. Values are means ± s.d. . Asterisks indicate that means differ from control samples, CrD samples cultured with medium alone and from CrD samples cultured with EC-LPS. *P<0.05. 2′,7′-dichlorodihydrofluorescein (DCF). (**C**) Caco-2 cells were treated for 24 h with butyrate and then were stimulated with EC-LPS for 4 h. (**C**, *left panel*) Immunoblot of p42/p44 phosphorylation. (**C**, *right panel*) Densitometric analysis of the band intensity. Values are means ± s.d., n = 6. β-actin was used as loading control for blot. (**D–E**) Confocal microscopy of phosphorylated p42/p44 (green) and number (**F**) of epithelial cells with phosphorylated p42/p44 per 100 epithelial in control (n = 10) and in CrD colonic mucosa (n = 14) before challenge (**D**) and after challenge with medium alone, medium with EC-LPS or EC-LPS with butyrate following 4 h of incubation(**E–F**). Nuclei counterstained with DAPI (blue). Scale bar, 10 µm. Values are means ± s.d.. Asterisks indicate that means differ from control samples, CrD samples cultured with medium alone and from CrD samples cultured with EC-LPS. *P<0.05.

RETRACTED

A pro-oxidative environment induces activation of different stress sensitive signalling pathways [31],[32],[33]. We demonstrated that butyrate prevented ROS-induced p42/p44 MAPK phosphorylation in LPS-stimulated intestinal epithelial cells. (Figure 2C). GSTA1/A2 siRNA antagonized the effect of butyrate in decreasing p42/p44 MAPK phosphorylation (Figure S2B).

We investigated the effect of butyrate in controlling ROS-induced p42p/44 MAPK phosphorylation in epithelia of CrD patients. Before challenge, higher p42/p44 MAPK phosphorylation was observed in CrD colonic mucosa compared with controls (Figure 2D). EC-LPS challenge led to an increase of p42/p44 MAPK phosphorylation at 4 h of incubation in CrD colonic mucosa but not in controls (Figure 2E and F). The increased expression of p42/p44 MAPK phosphorylation following EC-LPS challenge was efficiently controlled by butyrate (Figure 2E and F), which also reduced basal p42/p44 MAPK phosphorylation observed in the absence of any EC-LPS stimulation (Figure S3A and S3B).

### Butyrate decreases ROS mediated NF-κB activation and inflammatory response in intestinal epithelial Caco-2 cells upon challenge with LPS from *Escherichia Coli*

Since ROS levels enhance the signal transduction pathways for NF-κB activation in the cytoplasm and translocation into the nucleus, we examined whether butyrate is able to attenuate ROS-mediated NF-κB activation in Caco-2 cells challenged with EC-LPS. We demonstrated that butyrate was effective in controlling the translocation of phosphorylated p-65- NF-κB into nuclear extracts (Figure 3A) after 4 h and up to 24 h (data not shown) of challenge with EC-LPS. GSTA1/A2 siRNA antagonized the down-regulatory effect of the butyrate on phosphorylated p-65- NF-κB induced by EC-LPS (data not shown).

RETRACTED

**Figure 3:** Effect of butyrate on NF-κB activation and inflammatory response in intestinal epithelial cells challenged with LPS from *Escherichia Coli*. Caco-2 cells were treated for 24 h with butyrate and then were stimulated with EC-LPS for 4 h. (**A**) Immunoblot analysis of phospho-p65(Ser536) in cytoplasmic (*C*) and nuclear (*N*) cell fractions. αβ-tubulin and laminB were used as protein loading respectively for cytoplasmic and nuclear extract. (**B–C**) Caco-2 cells were treated for 24 h with butyrate and then were stimulated with EC-LPS for 24 h. (**B**, *left panel*) Immunoblot of COX-2 and ICAM-1. β-actin was used as loading control. (**B**, *right panel*) Densitometric analysis of the band intensity Values are means ± s.d., n = 6. Asterisks indicate that means differ from samples cultured with EC-LPS. *P<0.05. (**C**) TNF-α protein. Values are means ± s.d., n = 6. Asterisks indicate that means differ from samples cultured with EC-LPS. *P<0.05.

Since activation of the NF-κB/Rel transcription family plays a central role in inflammation through its ability to induce transcription of pro-inflammatory genes, we investigated whether butyrate is able to dampen down inflammatory response in Caco-2 cells challenged with EC-LPS. We showed that butyrate was effective in controlling COX-2, ICAM1 protein expression and TNF-α release induced by EC-LPS (Figure 3B and C). GSTA1/A2 siRNA antagonized the down-regulatory effect of the butyrate on COX-2, ICAM-1 protein levels and TNF-α release induced by EC-LPS (data not shown).

### Butyrate decreases ROS mediated NF-κB activation and mucosal inflammation in CrD mucosal epithelial cells upon challenge with LPS from *Escherichia Coli*

We investigated the effect of butyrate in controlling ROS mediated mucosal inflammation in CrD colonic mucosa. Before challenge, higher numbers of epithelial cells with p-65-nuclear localisation were observed in CrD colonic mucosa compared with controls (Figure 4 A). EC-LPS challenge led to an increase in numbers of epithelial cells with p-65-nuclear localisation at 4 h of incubation in CrD colonic mucosa but not in controls (Figure 4D). Moreover treatment of cultured biopsies with butyrate was highly effective in controlling EC-LPS induced p-65-nuclear localisation (Figure 4A).

RETRACTED

**Figure 4:** Effect of butyrate on mucosal inflammation in CrD mucosal epithelial cells challenged with LPS from *Escherichia Coli*. (**A**) Number of epithelial cells with p65 nuclear localisation per 100 epithelial cells in control (n = 10) and CrD colonic mucosa (n = 14) before challenge and after challenge with medium alone, medium with EC-LPS or EC-LPS with butyrate following 4 h of incubation. Nuclei counterstained with DAPI (blue). Scale bar, 10 µm. Values are means ± s.d.. Asterisks indicate that means differ from control samples, CrD samples cultured with medium alone and from CrD samples cultured with EC-LPS. *P<0.05. (**B**) Confocal microscopy of COX-2 (green) and ICAM-1(green) and number (**C**) of COX-2 and ICAM-1 positive lamina propria cells per mm^2^ of mucosa in CrD colonic mucosa (n = 14) after challenge with medium alone, medium with EC-LPS or EC-LPS with butyrate following 24 h of incubation. Nuclei counterstained with DAPI (blue). Scale bar, 10 µm. Values are means ± s.d., n = 14. Asterisks indicate that means differ from samples cultured with medium alone and from samples cultured with EC-LPS. *P<0.05. (**D**) TNF-α protein after challenge with medium alone, medium with EC-LPS or EC-LPS with butyrate following 24 h of incubation. Values are means ± s.d., n = 14. Asterisks indicate that means differ from samples cultured with medium alone and from samples cultured with EC-LPS. *P<0.05.

Butyrate also reduced the residual p65 localisation observed in CrD biopsies cultured in the absence of any EC- LPS stimulation (Figure S3C). To determine whether butyrate is able to switch off the mucosal inflammation in human EC-LPS stimulated CrD colonic mucosa, we also analysed the release of pro-inflammatory cytokines, such as TNF-α and COX-2 or ICAM-1 by mucosal mononuclear cells. This latter marker was studied as a broad factor of inflammation as described in previous study [28]. After 24 h of incubation, EC-LPS also induced an increase of ICAM-1 and COX-2 positive mononuclear cells and TNF-α release (Figure 4B, C and D) in CrD colonic mucosa compared with samples cultured in medium alone. The increased expression of ICAM-1, COX-2 and pro-inflammatory cytokine, as TNF-α release, following challenge with EC-LPS was efficiently controlled by butyrate (Figure 4B, C and D). Minimal TNF-α up-regulation and release, ICAM-1 and COX-2 were observed in controls after challenge with EC-LPS (data not shown).

## Discussion

This report describes the relationships among a bacterial product, oxidative stress and mucosal inflammation in the mucosa of patients with CrD. We have identified butyrate's role in intestinal epithelial homeostasis by promoting anti-oxidative responses and inhibiting mucosal inflammation in the colon of CrD patients.

RETRACTED

The short-chain fatty acid butyrate, which is mainly produced in the lumen of the large intestine by the fermentation of dietary fibers, plays a major role in the physiology of the colonic mucosa. It is also the major oxidative substrate for the colonocyte [34]. Impairment of IEC energy homeostasis is a typical feature of inflamed tissue in CrD. Constitutive energy expenditure mediated by persistent IEC activation and reduced energy supply may be the main causes of failure of IEC to preserve energy homeostasis [35].

Several studies report decreased butyrate oxidation in the inflamed mucosa of patients suffering from UC [36] or CrD [37] and in animal models of experimental colitis [38]. Although other studies found no defect in butyrate oxidation during IBD [39],[40],[41].

Previous studies in active IBD and in experimental DSS-colitis have shown that intestinal inflammation specifically affects butyrate metabolism [42],[43],[44]. Moreover, down-regulation of the Monocarboxylate Transporter 1 (MCT-1) is involved in butyrate deficiency in inflamed colonic mucosa of patients with IBD and of rats [45]. Thus, a decrease in MCT1 expression, which reduces the intracellular availability of butyrate [46] could affect not only its oxidation but also its cell regulatory effects.

Impaired energy availability as well as reduced tissue oxygen supply and the generation of intra and extracellular free radicals have also been to induce oxidative stress [47].

ROS are highly toxic to cells and oxygen radical formation in excess of physiological amounts may overtax the limited intestinal antioxidant defense system initiating oxidative injury to the gut [48] inducing damage to lipids, proteins and/or DNA. Moreover, increased oxidative stress has been seen to destroy the mucosal barrier of intestinal epithelial cells, increasing permeability. Different antioxidant defense mechanisms, including enzymatic antioxidant molecules, such as glutathione-S-transferase (GST) and non-enzymatic antioxidant molecules such as glutathione (GSH) are involved in protection against ROS. Deterioration of anti-oxidative glutathione metabolism [49] and increased colonic oxidative damage to proteins and DNA in association with impaired enzyme activity of Cu-Zn superoxide dismutase has been reported previously in patients with CrD [50]. Our studies demonstrate that butyrate was effective in controlling the increase of GSH reduced by EC-LPS in intestinal epithelial Caco-2 cell and in mucosal biopsies of CrD patients.

RETRACTED

There is limited evidence of butyrate's role in controlling oxidative stress in the colonic mucosa. In two in vitro studies, pre-treatment of isolated rat [51] or human [51] colonocytes with butyrate reduced H_2_O_2_-mediated DNA damage. Since the butyrate's antioxidant role is not primary, it may be secondary, influencing DNA repair systems and levels of enzymatic or non-enzymatic antioxidants. Fermentable fiber uptake in a rat model of TNBS-induced colitis [52] is reported to increase colonic concentrations of butyrate, to decrease colonic myeloperoxidase (MPO) activity and to restore colonic GSH concentration [53]. We demonstrated that butyrate was effective in controlling the decrease of GST-α protein levels and activity induced by LPS in intestinal epithelial Caco-2 cells and in mucosal biopsies of CrD patients. GST is a detoxifying enzyme system that provides defense against oxidative stress compounds [54]. Since oxidative stress induces the impairment of the intracellular ROS balance, we evaluated whether butyrate reduces ROS levels and ROS-mediated stress sensitive signalling pathways induced by EC-LPS in Caco-2 cells and in mucosal biopsies of CrD patients. We demonstrated that butyrate was effective in controlling the increase of ROS levels and reduces ROS-mediated p42/44 MAPK phosphorylation.

The most extensively studied intracellular pathway that is a target of ROS and oxidative stress is the transcription factor NF-κB [55]. NF-κB is found in cytoplasm and is bound to Iκ-Bα, which prevents it from entering the nuclei [56]. When these cells are stimulated, specific kinases phosphorylate Iκ-Bα, causing its rapid degradation by proteasomes [56]. Activation of NF-κB acts on genes for proinflammatory cytokines, chemokines (chemotactic cytokines that attract inflammatory cells to sites of inflammation) [56], enzymes that generate mediators of inflammation, immune receptors, and adhesion molecules that play a key role in the initial recruitment of leukocytes to sites of inflammation. Moreover, infiltrating macrophages and neutrophils that are abundantly present in inflamed gut expose the inflamed intestine to substantial oxidative stress by production of ROS [8] sustaining a vicious circle that leads to a progressive and uncontrolled inflammatory response. Our results demonstrate that butyrate controlled ROS-mediated p65 NF-κB activation in intestinal epithelial Caco-2 cells after challenge with LPS from *Escherichia Coli*. Since activation of the NF-κB/Rel transcription family plays a central role in inflammation through its ability to induce transcription of pro-inflammatory genes, we showed that butyrate decreases COX-2, ICAM1 protein expression and TNF-α release induced by EC-LPS.

RETRACTED

To provide the rationale and the proof-of-principle for using butyrate in CrD patients, we checked whether the mechanisms we observed in cell lines also take place in human CrD colons. Our approach to testing potential anti-inflammatory strategies in CrD, which we have used to study other inflammatory conditions and potential strategies to modulate the inflammatory response [12], is based on an *ex vivo* organ tissue culture model. This model represents a good approximation to in vivo studies since, all the anatomical connections in cultured biopsy tissues, are retained and all cell types (epithelial, myeloid, lymphoid) interact with neighboring cells within their natural environment. For this study we have used colonic mucosal biopsies which are routinely removed surgically.

We demonstrate that, in all CrD colonic tissues, butyrate reduced p65 phosphorylation and release of pro-inflammatory cytokines, such as TNF-α and COX-2 or ICAM-1 from mucosal mononuclear cells, thus restoring the pattern observed in controls after challenge with LPS from *Escherichia Coli*. Our study suggests that the restoration of intracellular ROS balance through appropriate control of the redox machinery may be a novel approach to treatment of CrD and may pave the way for the development of a new class of functional foods that, by enhancing butyrate production, could be effective treatments for CrD.

## Supporting Information

Figure S1 **Effect of butyrate on GST-α activity in EC-LPS stimulated intestinal epithelial cells and Crohn's mucosa.** (**A**) Intracellular GST catalytic enzyme activity was assessed by conjugation of chloro-2,4-dinitrobenzyne with reduced GSH. Asterisks indicate that means differ from samples cultured with medium alone and from samples cultured with EC-LPS. *P<0.05. (**B**) Caco-2 cells were transfected with either 50 nM human GSTA1/A2 siRNA or scrambled oligonucleotides and then challenged with butyrate for 24 hours. (**B**, *left panel*) Immunoblot of GST-α. β-actin was used as loading control. (**B**, *right panel*) Densitometric analysis of the band intensity. Values are means ± s.d., n = 6. (**C**) Intracellular GSH activity in butyrate treated CrD mucosal epithelial cells stimulated with EC-LPS. Asterisks indicate that means differ from samples cultured with medium alone and from samples cultured with EC-LPS. *P<0.05.
(EPS)

Figure S2 **Effect of butyrate on stress sensitive signalling pathways in EC-LPS stimulated intestinal epithelial cells.** Caco-2 cells were cultured with butyrate or transfected with either 50 nM human GST-A1/A2 siRNA or scrambled oligonucleotides and then challenged with EC-LPS. (**A**) Intracellular GSH levels. Asterisks indicate that means differ from samples cultured with medium alone and from samples cultured with EC-LPS. *P<0.05. (**B**, *left panel*) Immunoblot of p42/p44 phosphorylation in Caco-2 cells challenged with EC-LPS. β-actin was used as loading control. (**B**, *right panel*) Densitometric analysis of the band intensity. Values are means± s.d., n = 6. β-actin was used as loading control for blot.
(EPS)

Figure S3 **Expression of phosphorylated p42/p44-MAPk and p65-NF-κB in Crohn's mucosa.** Confocal microscopy of phosphorylated p42/p44 (green) (**A**) and number of epithelial cells (**B**) with phosphorylated p42/p44 per 100 epithelial in CrD colonic mucosa (n = 14) Nuclei counterstained with DAPI (blue). Scale bar, 10 µm. Values are means± s.d.. Asterisks indicate that means differ from CrD samples cultured with medium alone. *P<0.05. (**C**) Number of epithelial cells with p65 nuclear localisation per 100 epithelial in CrD colonic mucosa (n = 14). Nuclei counterstained with DAPI (blue). Scale bar, 10 µm. Values are means± s.d.. Asterisks indicate that means differ from CrD samples cultured with medium. *P<0.05.
(EPS)
